The article "The Therapeutic Potential of Wogonin Observed in Preclinical Studies" was retracted in 2023. Reasons: signs of a paper mill; compromised peer review; unreliable results or conclusions.

# The Therapeutic Potential of Wogonin Observed in Preclinical Studies

**DOI:** 10.1155/2021/9935451

**Published:** 2021-06-15

**Authors:** Javad Sharifi-Rad, Jesús Herrera-Bravo, Luis A. Salazar, Shabnum Shaheen, Seyed Abdulmajid Ayatollahi, Farzad Kobarfard, Muhammad Imran, Ali Imran, Luísa Custódio, María Dolores López, Mauricio Schoebitz, Miquel Martorell, Manoj Kumar, Hafiz Ansar Rasul Suleria, William C. Cho

**Affiliations:** ^1^Phytochemistry Research Center, Shahid Beheshti University of Medical Sciences, Tehran, Iran; ^2^Facultad de Medicina, Universidad del Azuay, Cuenca, Ecuador; ^3^Departamento de Ciencias Básicas, Facultad de Ciencias, Universidad Santo Tomas, Santiago, Chile; ^4^Center of Molecular Biology and Pharmacogenetics, Scientific and Technological Bioresource Nucleus, Universidad de La Frontera, Temuco 4811230, Chile; ^5^Department of Plant Sciences, LCWU, Lahore 54000, Pakistan; ^6^Department of Pharmacognosy and Biotechnology, School of Pharmacy, Shahid Beheshti University of Medical Sciences, Tehran, Iran; ^7^H.E.J. Research Institute of Chemistry, International Center for Chemical and Biological Sciences, University of Karachi, Karachi, Pakistan; ^8^Department of Medicinal Chemistry, School of Pharmacy, Shahid Beheshti University of Medical Sciences, Tehran, Iran; ^9^University Institute of Diet and Nutritional Sciences, Faculty of Allied Health Sciences, The University of Lahore, Lahore, Pakistan; ^10^Department of Food Science, Nutrition & Home Economics, Institute of Home and Food Sciences Government College University, Faisalabad, Pakistan; ^11^Centre of Marine Sciences, University of Algarve, Faculty of Sciences and Technology, Building 7, Campus of Gambelas, Faro 8005-139, Portugal; ^12^Department of Plant Production, Faculty of Agronomy, Universidad de Concepción, Avenida Vicente Mendez, 595, Chillán 3812120, Chile; ^13^Departamento de Suelos y Recursos Naturales, Facultad de Agronomía, Universidad de Concepción, Concepción, Chile; ^14^Department of Nutrition and Dietetics, Faculty of Pharmacy, and Centre for Healthy Living, University of Concepción, Concepción 4070386, Chile; ^15^Unidad de Desarrollo Tecnológico, Universidad de Concepción UDT, Concepción 4070386, Chile; ^16^Chemical and Biochemical Processing Division, ICAR–Central Institute for Research on Cotton Technology, Mumbai 400019, India; ^17^Department of Agriculture and Food Systems, The University of Melbourne, Melbourne 3010, Australia; ^18^Department of Clinical Oncology, Queen Elizabeth Hospital, Kowloon, Hong Kong

## Abstract

Wogonin is a flavonoid found in different plants such as roots of *Scutellaria baicalensis* Georgi distributed mainly in Asia and Europe. Dried root extracts of *S. baicalensis* with high content of wogonin, popularly known as “Huang-Qin” or Chinese or baical skullcap, have been used for long time in traditional Chinese medicine. Several health benefits are attributed to wogonin and derivatives showing anti-inflammatory, antiviral, anticancer, and antioxidant effects and more recently antineurodegenerative properties. Preclinical pharmacological activities of wogonin against diverse types of cancer such as breast, colorectal, and human gastric cancer will be presented in this review. In addition, studies on oxidative stress and bioavailability of wogonin will be discussed together with antineurodegenerative potential with special focus on Alzheimer's disease. Outcomes extracted from the last preclinical studies related to therapeutic applications of wogonin will be commented and updated in this review. The scientific evidence collected in this review aims to encourage transfer of the preclinical evidence of wogonin to new clinical studies.

The article "The Therapeutic Potential of Wogonin Observed in Preclinical Studies" was retracted in 2023. Reasons: signs of a paper mill; compromised peer review; unreliable results or conclusions.

## 1. Introduction

Flavonoids are polyphenolic secondary metabolites distributed naturally in seeds, fruits, stems, nuts, spices, pigments, vegetables, herbs, and flowers [1]. In human diet, the consumption of flavonoids is considered a phytonutrient, although some of these compounds can be chemically synthesized. Among these flavonoids, we find 5, 7-dihydroxy-8-methoxyflavone, a derivative of flavone, known as wogonin (Figure 1).

Wogonin was isolated and identified for the first time from *Scutellaria baicalensis* Georgi radix in 1930. *S. baicalensis* is a species of the Lamiaceae family distributed in the countries such as East Asia, North America, and Russia and in certain European places [2]. Wogonin is found in different parts of *S. baicalensis* such as roots [3] and whole herb [4] and different plants such as leaves of *Andrographis paniculata* (Burm.f.) Nees and stems of *Anodendron affine* (Hook. & Arn.) Druce [5]. In China, the dried root of *S. baicalensis* has been used as a medicinal plant for a long time and it is popularly known as “Huang-Qin” or Chinese or baical skullcap with a bitter taste. Dried *S. baicalensis* in traditional Chinese medicine have been described with curing properties on hepatitis, cirrhosis, jaundice, hepatoma, leukemia, hyperlipemia, atherosclerosis, and inflammatory diseases in China and Japan [6]. The extracts of this plant are marketed in different pharmaceutical forms such as tablets, drops, and capsules. Although wogonin is found most abundantly in *S. baicalensis*, the fact is that the yield is low and sometimes insufficient to achieve an industrial development. Hence, new ways to produce large amounts of wogonin are being studied [7]. Studies on *S. baicalensis* have identified wogonin, baicalein, baicalain, and wogonoside as the main active compounds of this plant, which imparts antioxidative properties and effectiveness in impeding the growth of cancer cells, showing its wider pharmacological potential [8–11]. These studies carried out both *in vitro* and *in vivo* on cells have provided a remarkable new approach to cancer prevention [12, 13]. A previous study has mentioned the anticancer properties of wogonin in different pathways, such as the upregulation of intracellular reactive oxygen species (ROS) production and p53 level, targeting phosphoinositide 3-kinase (PI3K/Akt) and mitogen-activated protein kinase (MAPK) pathways, inhibition of nuclear factor- (NF-) *κ*B, cell cycle arrest, and overcoming drug resistance [9]. Several studies show the potential role of phytochemicals in preventing drug resistance and sensitizing cancer cells to chemotherapeutic agents [14]. Other studies have also shown neuroprotective and anxiolytic effects of wogonin displaying an effect on central nervous system [8].

The article "The Therapeutic Potential of Wogonin Observed in Preclinical Studies" was retracted in 2023. Reasons: signs of a paper mill; compromised peer review; unreliable results or conclusions.

Despite all health benefits presented, some side effects must be revised and studied to be able to apply a safe range of dose. The main aim of this review is to report the preclinical pharmacological activities of wogonin and its bioavailability.

## 2. Preclinical Pharmacological Activities of Wogonin

### 2.1. Anticancer Activity

As described previously, wogonin displays several important biological properties highly relevant to human health improvement. Probably, the most explored are its antitumor features; it strongly induces apoptosis of different cancer cells, including leukemia, multiple myeloma, lymphoma, and ovarian cancer [9, 15–21]. Wogonin supplementation has been proved effectual against different breast cancer cell lines like triple-negative breast cancer (TNBC) and its allied cell lines, i.e., BT-549 and MDA-MB-231, owing to its effect on cell viability and cell proliferation. Furthermore, cell cycle of cancer cell lines is detained by halting the expressions of cyclin D1, cyclin B1, and cyclin dependent kinase 1 (CDK1), apoptosis induction, and enhancement in Bax/Bcl-2 (B-cell lymphoma 2) ratio and caspase-3 cleavage, with these noticeable mechanistic routes being related to anticancer ability of wogonin [22].  Figure 2 summarizes anticancer activity of wogonin.

The wogonin administration against human gastric cancer cells (SGC-7901) and human lung adenocarcinoma cells (A549) caused dose-dependent inhibition in cell proliferation and induced apoptosis. The wogonin caused the significant change in the morphology of the cell and expression of key enzymes involved in the glycolysis and tricarboxylic acid cycle. In case of human gastric cancer cells SGC-7901 wogonin treatment showed potent reduction in the activities of lactate dehydrogenase (LDH) and succinate dehydrogenase (SDH) and lowered the generation of adenosine triphosphate (ATP) as compared to control. However, in A549 cells, wogonin had no effect on kinase activity but significantly reduced the LDH activity. The significant decrease in hypoxia-inducible factor- (HIF-) 1*α* and monocarboxylate transporter- (MCT-) 4 protein expression has also been observed in SGC-7901 cells, but not in A549 cells. The outcomes of the findings revealed the role of wogonin in energy inhibition, cell proliferation, and downregulating the HIF-1*α* and MCT-4 expression [23]. In another study, wogonin showed *in vitro* antiproliferative activity against A549 and HeLa cancer cell lines [24]. In addition, the authors of this study conjugated wogonin with a fluorophore and observed that wogonin acts at mitochondrion to exerts its pharmacological function.

The article "The Therapeutic Potential of Wogonin Observed in Preclinical Studies" was retracted in 2023. Reasons: signs of a paper mill; compromised peer review; unreliable results or conclusions.

The role of wogonin against colorectal cancer (CRC) has not yet been fully established. However, the outcomes of a preclinical study displayed that wogonin treatment induces apoptosis in human CRC HCT-116 cell by accelerating the endoplasmic reticulum (ER) stress by localization of p53 through activation of phosphor-p53 [21]. Moreover wogonin has been seen inhibiting the tumor angiogenesis through the degradation of HIF-1*α* [25], inhibiting the proliferation of human CRC cells when introducing autophagy, apoptosis, and cell cycle arrest at G2/M through the modulation of the marking PI3K/AKT and signal transducer and activator of transcription (STAT3) [26]. Persistent STAT3 activation promotes chronic inflammation and increases susceptibility of healthy cells to carcinogenesis [27]. It has been also seen activating different ways through molecular targets to perform anticarcinogenic effects [28]. Likewise, in HT-29 cells, wogonin induced the phosphorylation and acetylation of p53 by inhibiting the activities of mouse double minute 2 homolog (MDM2). Additionally, reduction in glycolysis of transplanted wild-type p53 expressing A2780 cells on nude mice is also observed through wogonin supplementation [29]. Wogonin supplementation has been reported to reduce the invasiveness of MDA-MB-231 cell by inhibiting the lipopolysaccharide (LPS) activities and synthesis of interleukin- (IL-) 8 and matrix metallopeptidase-9 (MMP-9). It reduces the leukotriene B4 receptor 2 (BLT2) through inhibition of 5-lipoxygenase (5-LO) [30].

The possible wogonin administration against chronic rhinosinusitis (CRS) with nasal polyps (CRSwNP) has been *in vitro* studied with special reference to evaluate its apoptosis induction role. Purposely, double immunofluorescence, immunohistochemistry, flow cytometry, and immunoblotting were carried out. Resultantly, the elevated expression of HIF-1*α* and survivin in tissues obtained from eosinophilic patients with CRS was downregulated by the supplementation of wogonin [31]. Earlier, Hong et al. [32] carried out a research to explore the role of wogonin in cancer cell migration and invasion. These authors provided the *in vitro* supplementation of wogonin with concentration of 50–100 *μ*M and observed significant inhibition in the MHCC97 L and PLC/PRF/5 cells migration and invasion alongside MMP-9 activity reduction [32]. More potent effect of wogonin against cancer cell viability and proliferation is evident when this compound is combined with other phytochemicals. For example, the combination of oxaliplatin and wogonin elucidated promising reduction in cell viability of BGC-823 cells of zebrafish xenograft model through modulation of phospho-ULK1 (Ser555) and phospho-JNK (Thr183/Tyr185) expressions [33].

The article "The Therapeutic Potential of Wogonin Observed in Preclinical Studies" was retracted in 2023. Reasons: signs of a paper mill; compromised peer review; unreliable results or conclusions.

The intraperitoneal administration of wogonin at concentrations of 10 and 20 mg/kg in rats improves the histological and functional anomalies. Furthermore, it inhibits IL-6, tumor necrosis factor- (TNF-) *α*, IL-1*β*, and phosphorylation of p38 MAPK [34]. The oral administration of wogonin caused significant inhibition of the etoposide-induced oxidative DNA damage and apoptosis; however, effect was produced as a function of wogonin concentration. The etoposide caused DNA mutation after downregulating the expression of 8-oxoguanine glycosylase (OGG1) repair gene alongside enhancement in 8-hydroxydeoxyguanosine (8-OHdG) DNA damage marker, lipid peroxidation, and inhibition of antioxidant enzymes. However, the wogonin caused rectification of these anomalies, thus helpful to control DNA damage [35]. In addition, wogonin-induced ROS block TNF-induced NF-*κ*B activation through the inhibition of NF-*κ*B p65 subunit phosphorylation and consequently the DNA binding of NF-*κ*B [36]. The aberrant activation of NF-*κ*B involves aggressive tumor growth and resistance to therapeutic treatment [37], so this modulation by wogonin may exert an important role in tumor progression.

The wogonin supplementation caused marked decline in the expression of serum osteopontin (OPN) levels in 3T3-L1 adipocytes of mice. Further it improved the peroxisome proliferator-activated receptor alpha (PPAR-*α*) expression and activity alongside reduction of c-Fos and phosphorylated c-Jun level. It is also reported that the wogonin addition caused reduction in p38 MAPK phosphorylation by its specific inhibitor SB203580 and thus enhanced the PPAR-*α* activity and reduced OPN expression [38].

The article "The Therapeutic Potential of Wogonin Observed in Preclinical Studies" was retracted in 2023. Reasons: signs of a paper mill; compromised peer review; unreliable results or conclusions.

Among the major mechanistic concerns are wogonin inhibitory effect on upstream signaling of peroxisome PPAR-*γ* and CCAAT/enhancer binding protein- (C/EBP-) *β* expression and inhibition of the adipocyte differentiation through effecting the PPAR-*γ*, C/EBP-*α*, and C/EBP-*β* in 3T3-L1 preadipocytes. Moreover, wogonin significantly reduced the phosphorylation of Raf/extracellular mitogen-activated protein kinase 1 (MEK1)/signal-regulated protein kinase 1/2 [39]. In case of liver cancer, the wogonin supplementation is reported to decrease the cell viability of RAW264.7 cells through declining the cytokines like IL-6 and TNF-*α* responses and suppressing the PPAR-*γ*-meditated phosphorylation [40]. Wogonin also exhibits *in vitro* and *in vivo* synergistic effects with other chemotherapeutic drugs, such as etoposide and paclitaxel, and acts as a chemosensitizer; i.e., it is able to revert drug resistance of tumors [18, 41, 42]. Its antitumoral efficacy was confirmed by *in vivo* studies, therefore opening the possibility of clinic uses [29, 43–46].

### 2.2. Antineurodegenerative Activity

Globally, Alzheimer's disease (AD) is recognized as a major neurodegenerative disorder. The accumulation of intrinsically disordered protein, amyloid beta (A*β*) (A*β*_40_ and A*β*_42_) and tau, is considered as a leading cause of this disease. However, wogonin supplementation has the ability to uplift the A*β* removal in the primary neural astrocytes. Moreover, it inhibits the glycogen synthase kinase 3 beta (GSK3*β*) via mammalian target of rapamycin (mTOR) inhibition, thus inhibiting the tau phosphorylation in primary neural astrocytes [47]. Similar observations were made by Huang et al. [48]. These authors noticed the improved clearance of A*β*_40_ and A*β*_42_ and tau after oral treatment of wogonin in the performance of triple transgenic AD mice on the Morris water maze, Y-maze, and novel object recognition, alongside increasing the neurite length and complexity of Tet-On A*β*_42_-GFP SH-SY5Y neuroblastoma cells.  Figure 3 summarizes neuroprotective effect of wogonin.

The wogonin also has the positive impact on bone marrow stem cells (BMSCs) health by promoting the retinal neuron-like differentiation. It also diminishes the stem cell markers expressions and reduces the mature retinal neurons markers, photoreceptors, and bipolar cells [49].

ER stress has been involved in the pathogenesis of many oncogenic events and initiates many neurodegeneration problems. The wogonin proved effectual in reducing the ER stress in rat dorsal root ganglion (DRG) neurons by decreasing the number of the terminal deoxynucleotidyl transferase dUTP nick end labeling- (TUNEL-) positive DRG neurons and increased expression of superoxide dismutase [20] and reduction in malondialdehyde (MDA) level. It was further reported to induce apoptosis by lowering the level of Bax, accelerating the Bcl-2 level, and downregulating the ER stress genes and phosphorylation of pancreatic ER stress kinase (PERK) and eukaryotic initiation factor 2 alpha (eIF2*α*) [50]. In glioma cells, wogonin promoted apoptosis by upregulating Bad gene expression and cleaved caspase-3 gene activation and by downregulating Bcl-2 expression [51]. ER stress reducing effect of wogonin has been further documented in the outcomes of Xu et al. [52]. These authors observed reduced ER stress by downregulating the glucose-regulated protein 78 (GRP78), GRP94, C/EBP-homologous protein, active caspases 3 and 12, phosphorylation of PERK, and eukaryotic initiation factor 2 alpha (eIF2*α*). TNF inhibition behavior of wogonin is also well established. Mechanistically, wogonin increases the partial thromboplastin time and prothrombin time and suppressing the thrombin-catalyzed fibrin polymerization [53].

The article "The Therapeutic Potential of Wogonin Observed in Preclinical Studies" was retracted in 2023. Reasons: signs of a paper mill; compromised peer review; unreliable results or conclusions.

Intervertebral disc degeneration (IVDD) results through the loss of the extracellular matrix in the local nucleus pulposus region. Wogonin reduced the inflammatory responses like IL-1*β*-induced inflammatory mediators, i.e., inducible nitric oxide synthase (iNOS), IL-6, and cyclooxygenase 2 (COX2) with upregulation of collagen II and activation of nuclear factor erythroid 2-related factor 2 (Nrf2)/heme oxygenase-1 (HO-1), superoxide dismutase 2 (SOD2), NAD(P)H quinone dehydrogenase 1 (NQO1), glutamate-cysteine ligase catalytic subunit (GCLC) (Nrf2/HO-1-SOD2-NQO1-GCLC) signaling axis [54–57], and prostaglandin E2 production [58–60].

### 2.3. Other Biological Activities

Besides antitumoral and neuroprotective activities, wogonin also displays antiviral (anti-hepatitis B virus, HBV), antioxidant, and chondroprotective properties [9, 11, 20, 61–64]. Furthermore, wogonin displays anxiolytic properties in a mice model, without exhibiting the characteristic sedative and muscle-relaxing properties of benzodiazepines [3], and has anticonvulsant effects [65]. The 5, 7-dihydroxyl groups of wogonin chemical structure seem to be responsible for benzodiazepine binding site, which crucially regulates the anxiolytic property of wogonin [66]. In a recent study, wogonin exhibited antifibrotic effect on a mice model, being suggested as a possible therapeutical strategy to treat and prevent liver fibrosis [67]. To the best of our knowledge, no clinical trials have been reported on wogonin.

The article "The Therapeutic Potential of Wogonin Observed in Preclinical Studies" was retracted in 2023. Reasons: signs of a paper mill; compromised peer review; unreliable results or conclusions.

## 3. Bioavailability of Wogonin

The evidence of wogonin *in vitro* effects has been increasing in the last years; however, the transfer of this result *in vivo* is poorly registered. A study performed in Sprague Dawley rats determined that the intragastric plasmatic levels of wogonin reached the peak in 28 min after administrating 100 mg/kg with a maximum concentration (*C*_max_) of 300 ng/mL [46]. Moreover, after an intravenous administration of 20 mg/kg, wogonin was detected in many tissues including testicles, brain, and heart, while the highest levels were detected in kidneys and liver with a low wogonin bioavailability to 1.1% [46]. Similarly, Tsai et al. [68] accounted that there was a rapid increase in its plasmatic level followed by a retarded elimination rate after the intravenous administration of 5 mg/kg of wogonin in Sprague Dawley rats. Another study investigated the pharmacokinetic characteristics of wogonin in Sprague Dawley rats' plasma after the oral administration of the *S. baicalensis* extract. The research revealed that 4.5 g of extract per kg of weight had a *C*_max_ 79.8 ng/mL in a *T*_max_ of 15 min and a slow elimination of 170.4 compared with other flavonoids found in the same extract [69]. Another study evaluated the bioavailability in rats' plasma after the oral administration of 5 components that come from different sources; wogonin revealed that *T*_max_, *C*_max_, and T_1/2_ were 5.28 h, 193.3 *µ*g/L, and 38.7 h, respectively [70]. Additionally, bioavailability of wogonin combined with docetaxel has been measured in rats' plasma stating that after the oral administration of 40 mg/kg of wogonin its *T*_max_ was 0.58 h, while the *C*_max_ and T_1/2_ were 76.8 ng/mL and 2 h, respectively [71]. As observed, wogonin has a very low bioavailability when administered alone; however, an improvement in its bioavailability has been registered when administered in combination with other components. A former research established that, after the administration of a *Scutellaria barbata* D.Don extract, the free form of wogonin was present with a *C*_max_ of 16.1 ng/mL, and when administered in combination with other metabolites the wogonin concentration in rats' plasma doubled [72].

The oral administration is still an efficient route to administer medicine, especially for chronic diseases which need long-term treatment and when patients do not accept intravenous administration, even though the solubility of some drugs makes their bioavailability low when administered this way. In addition, many of the results showing the biological activities of wogonin have been generated *in vitro* because the main limitation of this powerful phytochemical is its low solubility in water, having a direct impact on its bioavailability, therefore limiting its application. However, wogonoside (glycosylated form of wogonin) has high plasma concentration and bioavailability after oral administration in rats [73]. So, developing methods to improve wogonin solubility and liberation appears to be an essential task to make *in vivo* use of this powerful molecule. Nowadays, with the development of some techniques, the preparation of wogonin exhibits a better absorption and major bioavailability. A study evaluated the effect of the wogonin charge in a solid lipidic nanoparticle of breast cancer (MCF-7), providing evidence of a prolonged cytotoxic effect in concentrations of 200 *µ*M [74], proposing an efficient strategy to improve its bioavailability and liberation. Another study performed in 6 Beagle dogs informed that solid dispersion technology is a good strategy to improve wogonin solubility, showing evidence of a *C*_max_ of 7.9 *µ*g/L, a *T*_max_ of 0.3 h, a T_1/2_ 5.1 h, and absolute bioavailability of 4%. This data reveals substantial improvement when compared to the administration of raw compound [75]. Micelles of Zeina-lactoferrin have reflected a high efficiency in the liberation of wogonin. In this study, the self-assembled micelles formed by corn protein, Zeina, as hydrophobic nucleus chemically combined with lactoferrin could coencapsulate rapamycin and wogonin improving their bioavailability when they are parent administered [76]. Another study that developed wogonin liposomes modified with glycyrrhetinic acid for an intended use in therapy against cancer exhibited improvement in the biodistribution, accumulation, and therapeutic efficacy [77].

The article "The Therapeutic Potential of Wogonin Observed in Preclinical Studies" was retracted in 2023. Reasons: signs of a paper mill; compromised peer review; unreliable results or conclusions.

## 4. Conclusions

Recently, seek of new bioactive compounds and development of new drugs has been focusing on natural products such as flavonoids. Wogonin is a flavonoid that has been studied and used for long time in Chinese medicine and it can be found as tablets, drops, or capsules. Beneficial properties on health have been demonstrated throughout the manuscript in either cancer treatments, neuroprotective potential, and antioxidative effect. The mechanisms of wogonin described as anticancer include serine-threonine kinase and AMP-activated protein kinase pathways and p53-dependent/independent apoptosis. In addition, its antineurodegenerative potential is remarkable since wogonin supplementation has the ability to uplift the A*β* removal in the primary neural astrocytes and inhibit the GSK3*β* via mTOR inhibition, thus inhibiting the tau phosphorylation in primary neural astrocytes.

Obtained results for wogonin, in terms of, for example, antitumoral, neuroprotective, anti-inflammatory, and antiviral activity, stress its efficacy and safety and encourage further work aiming at its translation into clinical drugs. However, to the best of our knowledge, no clinical trials have been conducted so far, on this molecule. The scientific evidence reported in this review aims to encourage the development of new clinical evidence that studies the therapeutic effect of wogonin, enriched extracts of the compound, or enriched herbal treatments that report adequately its phytocomposition. The oral bioavailability of wogonin is low and bioavailability enhancement through nanotechnology tools will allow taking a better profit of its potential benefits on human health. Nevertheless, despite all therapeutic potential, all new drugs require to be studied in depth, even natural ones, since it could present also side effects such as effects of high dosage and long-term use. In addition, a better understanding of mechanisms involved in the biological activities of wogonin is needed. Hence, the development of new formulations to achieve a successful administration of wogonin should be considered, focusing on target, drug release, and design of nano-microparticles which are necessary in clinical trials.

The article "The Therapeutic Potential of Wogonin Observed in Preclinical Studies" was retracted in 2023. Reasons: signs of a paper mill; compromised peer review; unreliable results or conclusions.

## Figures and Tables

**Figure 1:** Source and chemical structure of wogonin.

**Figure 2:** Anticancer activity of wogonin (a) in breast cancer cell lines (TNBC), (b) in gastric cancer cell lines (SGC-7901), and (c) in colorectal cancer cell lines (CRC HCT-116). Wogonin acts as anticancer agent mainly by inhibiting the cell cycle through downregulating cyclins and inducing apoptosis in the cancerous cells.

**Figure 3:** Neuroprotective effect of wogonin. Wogonin inhibits the glycogen synthase kinase 3 beta (GSK3*β*) via mammalian target of rapamycin (mTOR) inhibition, thus inhibiting the tau phosphorylation in primary neural astrocytes.
